The article "Genistein: Therapeutic and Preventive Effects, Mechanisms, and Clinical Application in Digestive Tract Tumor" was published in 2022. Journal: Evid Based Complement Alternat Med.

# Genistein: Therapeutic and Preventive Effects, Mechanisms, and Clinical Application in Digestive Tract Tumor

**DOI:** 10.1155/2022/5957378

**Published:** 2022-06-29

**Authors:** Shenglin Hou

**Affiliations:** School of Pharmacy, Nanjing University of Chinese Medicine, Nanjing, China

## Abstract

Genistein is one of the numerous recognized isoflavones that may be found in a variety of soybeans and soy products, including tofu and tofu products. The chemical name for genistein is 4′, 5, 7-trihydroxyisoflavone, and it is found in plants. In recent years, the scientific world has become more interested in genistein because of its possible therapeutic effects on many forms of cancer. It has been widely investigated for its anticancer properties. The discovery of genistein's mechanism of action indicates its potential for apoptosis induction and cell cycle arrest in gastrointestinal cancer, especially gastric and colorectal cancer. Genistein's pharmacological activities as determined by the experimental studies presented in this review lend support to its use in the treatment of gastrointestinal cancer; however, additional research is needed in the future to determine its efficacy, safety, and the potential for using nanotechnology to increase bioavailability and therapeutic efficacy.

## 1. Introduction

One of the main purposes of scientific study nowadays, due to the growth in life expectancy, is to prevent the start of disorders related to age. Although heredity is recognized to have a role in lifestyle, specifically dietary habits and physical activity have been proved to show the main role at the beginning of certain illnesses [1, 2]. In this regard, functional foods and the nutraceutical area have recently attracted increased interest Salehi et al. [3, 4]. Latterly, in particular, it leads to the creation of plant extracts-based products and/or bioactive compounds isolated with well-known and, over time, increasingly detailed biological capabilities [5, 6]. In the year 2018, the estimated new cases of gastrointestinal (GI) were 4.80 million and worldwide related deaths were 3.40 million. Of the global cancer incidence, GI cancers account for 26% and 35% of all cancer-related deaths [7].

## 2. Review Methodology

In the current paper literature review was carried out by scouring the scientific databases, i.e., PubMed, Google Scholar, and Scientific approach in the most relevant material. Genistein, pharmacology, molecule mechanisms, bioavailability, and clinical studies were the search terms. For a competent evaluation, the selected articles were thoroughly examined. *In vivo* and *in vitro* experimental pharmacologic research on substances and extracts from plants, as well as the types of preclinical trials, dosages, and concentrations on which pharmacologic features, pathways, and genistein action's molecular targets, was assessed. The most relevant clinical trials were included. PubChem and SciFinder were used to validate compound structures. The Plant List (https://www.theplantlist.org) was used to determine the plants' scientific names.

The article "Genistein: Therapeutic and Preventive Effects, Mechanisms, and Clinical Application in Digestive Tract Tumor" was published in 2022. Journal: Evid Based Complement Alternat Med.

### 2.1. Genistein and Sources

Soy foods include soy cheese and soy drinks, which are the best-known genistein sources (soy-based brews and soy milk). Genistein's level in the ripe soybeans range varies with an average range of 81 mg/100 g frequently used for comparison [8]. Soy foods also include daidzein, a significant isoflavone that varies from genistein in that it lacks the hydroxyl group (OH^−^) at the fifth position compared to genistein. Both isoflavones can be found as aglycones or glycosides. The derivatives O-b-d-glucoside in genistein and daidzein are the most frequent glycoside forms. Because soy is used in so many traditional Asian dishes, in Asian countries, the average nutritional isoflavone intake varies from 25 to 50 mg/d. The estimated intake in the West is much low than in Asia [9, 10].

The second most abundant genistein source is legumes, which have a concentration of 0.20–0.60 mg/100 g and daidzein, a closely related isoflavone [11]. An example of a legume is the genus Lupinus (often referred to as lupin), which is generally farmed for its seeds, having a dietary value comparable to soybean. Considerable levels of genistein are found in broad beans and chickpeas, though not as much in soybeans. With an assessed range of 0.03–0.2 mg/100 g, the amount of genistein found in fruits, vegetables, and nuts differs greatly [12]. However, genistein amounts of up to 4.4 mg/100 g have been found in a few Hungarian instinctive cherry cultivars. Several databases [8] have an extensive list of foods with their genistein concentration. The most frequent strategy for improving the nutritional and therapeutic qualities of specific foods is to utilize a biotechnological approach to enhance isoflavonoid output by sprouting seeds. Seed germination metabolic processes have been revealed to improve dietary value by increasing the plant's secondary metabolites (isoflavonoids) and vitamin contents [13–17]. As a result, genistein's high content and further isoflavonoid aglycones in germinated soybean seeds and correlated products have been thoroughly reported [18]. During the fermentation process of soybean products, the amount of genistein and interrelated aglycones increases [19]. From nonlegume plants to obtain genistein, i.e., rice through genetic manipulation is also possible. By cloning process, the enzyme IFS from a genistein-rich soybean cultivar transgenic rice line with 30 folds more genistein contents was formed [20]. Latterly replacing soy-based meat, soy cheese, soy milk, and soy-yogurt has acquired famous in the United States and Europe, thanks to the medical significance of genistein and related isoflavonoids [21].

The article "Genistein: Therapeutic and Preventive Effects, Mechanisms, and Clinical Application in Digestive Tract Tumor" was published in 2022. Journal: Evid Based Complement Alternat Med.

### 2.2. Genistein's Chemical Synthesis

Synthesis of isoflavone remains a crucial auxiliary in the traditional logic of structural explanation of natural analogs. Because of the ease with which isoflavones may be converted into most other kinds of isoflavonoids, they are usually the first synthetic targets. Currently, the importance of synthetic procedures has transferred progressively to report the requirements of the biology–chemistry interface, such as enantiopure derivative's stereoselective synthesis such as isoflavone-epoxides [22], isoflavones [23], isoflavones [24], and pterocarpans. The chalcone and deoxybenzoin (2-hydroxyphenyl benzyl-ketone) procedures are the two traditional methods for making isoflavones. Other methods, such as flavanone rearrangement, chalcone epoxide rearrangement, and cyclization, palladium-catalyzed organolead facilitated arylation of chroman-4-ones, cross-coupling of 3-halochromones with aryl boronic acids, and so on, are fewer common and have been studied by [25]. In a deoxybenzoin method, the base-catalyzed condensation of the 2-hydroxyphenyl benzyl-ketone with a reagent containing an activated C1 unit is used. Recently, this method is widely used, employing a wide range of C1 reagents in many reaction circumstances. Its value is proven in Scheme 1 [25] for recent genistein (1) synthesis. Deoxy-benzoin (9), obtained through Houben Hoesch acylation of phloroglucinol (7) with p-hydroxyphenyl acetonitrile (8), treatment with [(Me2N+14CHCl) Cl], formed in situ via reacting PCl5 and N, N-dimethylformamide (DMF), to yield 90% genistein. More yield of this might be utilized in a “one-pot” procedure under mild circumstances and can be scaled up to tone volumes. Schemes 1 and 2 show the synthesis of genistein.

### 2.3. Bioavailability and Safety of Genistein

Genistein in its free form from soy extracts has been demonstrated to be highly accessible in a variety of experimental scenarios, including *in vivo* experiments. In portal vein plasma, genistein was quickly accessible and detectable 15 minutes afterwards treatment in easily moving rats (unanesthetized) by using a cannula in the portal vein, through AUC standards (0–24 h) of 54 for genistein [27]. The fact that genistein has a low water solubility limits its bioavailability following oral administration [28]. Genistein has also a bitter taste [29], so new formulations are needed to address both the bioavailability and the acceptable flavor issues. Both people and experimental animals have shown that genistein undergoes extensive metabolism in the gut and after absorption. Di-hydrogenistein, sulfate conjugates of genistein, and also their metabolites are found in excreta and the blood. The gut microbiota, yielding 2-(4-hydroxyphenyl)propionic acid and di-hydrogenistein is best known to be cleaved the C ring of the isoflavonoid skeleton [30–32]. For conjugation, the 3 OH groups (5, 7, and 4′) are often existing although the genistein 7-glucuronide-4′-sulfate and genistein 4′, 7 di-glucuronide by-products are predominant metabolites in plasma [33].

The article "Genistein: Therapeutic and Preventive Effects, Mechanisms, and Clinical Application in Digestive Tract Tumor" was published in 2022. Journal: Evid Based Complement Alternat Med.

Various complicated effects of these compounds suggest that high quantity injection of isoflavones might cause detrimental effects; there is no strong evidence that consuming high quantity of isoflavones in the diet is detrimental to people [34]. However, at a single dosage that crosses average nutritional consumptions of pure unconjugated isoflavones, there was negligible clinical harm in strong postmenopausal females [35]. Anticancer drugs' genotoxicity, such as genistein, may be advantageous since it promotes the death of cancerous cells through apoptosis and other cytotoxic ways. Normal cells, on the other hand, would be negatively affected by these chemicals. *In vitro* and in experimental animals, genistein has been shown to have potentially harmful effects (apoptosis, cell growth suppression, DNA damage, and topoisomerase inhibition) and genotoxic [36–39]. However, the concentrations of genistein employed in these trials were substantially greater than the physiologically related amounts achieved via consuming soy foods or supplements by dietary or pharmacologic means. *In vivo* studies, on the other hand, consistently yielded negative genotoxicity data [40]. Pure genistein administration to postmenopausal women aged 46–68 years revealed low toxicity at dosages of 16 mg genistein/kg body weight [35].

On fertility and fetus development, the effects of genistein have received high attention. In a rat model, clinically relevant dosages of genistein were found to have significant deleterious effects on the estrous cycle, ovarian differentiation, and fertility [41]. During uterine development, exposure to genistein induced various negative impacts in animal models, according to research [41, 42]. The contradictory results are most likely due to discrepancies in exposure time, dosages, and experimental endpoints. Human fetuses' exposure to isoflavones during their development in the uterus as well as during infancy through breast milk may possible [43]. In soy formula-fed newborns, the amounts of genistein range from 10-  to > 100-fold higher than in the wide-ranging population [44]. These doses can raise blood genistein levels to levels that are consistent with significant biological estrogenic effects in children. However, there is a dearth of evidence from human trials; thus, future research about the effects of genistein on human fertility and/or fetal growth is needed.

The article "Genistein: Therapeutic and Preventive Effects, Mechanisms, and Clinical Application in Digestive Tract Tumor" was published in 2022. Journal: Evid Based Complement Alternat Med.

### 2.4. Nanotechnology Increases Genistein Bioavalibility and Saftey

Encapsulated genistein can be used to administer colloidal drugs for cancer treatment. A study carried out a hemolysis experiment and discovered that genistein-loaded poly(lactic acid) nanoparticles were nontoxic [45]. Genistein potentiated its antiproliferative and antioxidant effects on HT29 human colon cancer cells after encapsulation with PEGylated silica nanoparticles by modulating endogenous antioxidant enzymes and H_2_O_2_ production, simultaneously activating apoptosis and autophagy, unlike free genistein, which only activates apoptosis in a lower proportion [46, 47]. Nanotechnology is often regarded as the most significant engineering breakthrough since the industrial revolution. Biodegradable polymer nanoparticles can deliver drugs in a regulated and targeted manner, with improved efficacy and fewer side effects [48]. MTT tests on aggressive prostate cancer cell lines verified genistein-gold nanoparticles conjugates in vitro. The stability and bioactivity of genistein-gold nanoparticles as an antioxidant and antiprostate cancer agent, as well as minimal toxicity against human primary cells, are indicated by cytotoxicity and IC50 analyses [49]. To obtain increased antitumor activity in U87MG human glioblastoma cells, temozolomide and genistein dual-drug-loaded poly(lactic-co-glycolic-acid) nanoparticle systems (Gen-TMZ-NPs) were designed. According to the findings of a study, Gen-TMZ-NPs had increased antitumor activity in U87MG cells [50].

### 2.5. Genistein Anti-Cancer Activity

Like Genistein, other similar isoflavones can block cell development/the formation of malignancies in the prostate, stomach, blood, bladder, and lungs. Biochanin A and genistein are appeared to prevent *in vitro* the division of human stomach cancer cell lines via stimulating a signal-transduction mechanism that is responsible for apoptosis [51]. Not genistein but biochanin A dramatically suppressed tumor development when these cancerous cells were put into mice. Genistein suppresses the proliferation of leukemia cells when linked to a monoclonal antibody, and a derivative of prenyl-isoflavone has been settled for acute leukemias as oral treatment [52].  Table 1 summarizes the genistein used to treat cancers other than gastrointestinal cancer.  Figure 1shows the anticancer effect of genistein by regulating different pathways.

The article "Genistein: Therapeutic and Preventive Effects, Mechanisms, and Clinical Application in Digestive Tract Tumor" was published in 2022. Journal: Evid Based Complement Alternat Med.

### 2.6. Mechanisms and Clinical Application of Genistein in Gastric Cancer

#### 2.6.1. Epidemiologic Data

From an interventional standpoint, in preventing stomach cancer, the part of soybean products is controversial. In the Korean Multicenter Cancer Cohort, a nested case–control approach recommended that a high serum concentration of isoflavone was linked to a less hazard of gastric cancer [72]; however, in the Japan Public Health Center-Based Prospective Approach, a parallel nested case–control study has shown no link in gastric cancer and isoflavone ingestion among Japanese women and men [72, 73].

#### 2.6.2. *In Vitro* Studies

In the case of primary gastric cancer cells (20 M for 24–72 h) in preclinical models, genistein can cause apoptosis by upregulating the proapoptotic protein Bcl2-related X protein (Bax) expression and downregulating the antiapoptotic protein B-cell lymphoma2 (Bcl2) [74]. Genistein's different concentrations having apoptosis causing ability in SG-7901 transplanted cells in the subcutaneous tissue of nude mice was thought to be due to a comparable change in the Bcl2 and Bax ratio [75]. Genistein therapy caused apoptosis in the human stomach cancer cell line BGC-823 in a time and dose-dependent way and decreased the cell growth. On transcription factor NFB activation in this model, the compound had a strong inhibition effect resulting in a decrease in cyclooxygenase 2 (COX2) protein quantities [76].

In BGC823 cells and SGC7901, genistein's capacity to induce G2/M to stop the cell cycle was investigated. By upregulating phosphatase and tensin homolog, genistein (20–80 M) reduced Akt activation (PTEN) [77]. To examine the anticancer processes of the drug and to discover the genistein-regulated components, researchers used a stable isotope labeling in combination with amino acids in the cell culture quantitative proteomics method. The expression of 86 proteins involved in regulating the process of G2/M transition, proliferation, and growth of the cell was modified by genistein in SGC7901 cells treated with 40 M genistein for about 48 hours, with 49 upregulated and 37 downregulated proteins [78].

A subpopulation of tumor cells, and Gastric cancer stem cells (GCSCs) having the self-renovation ability and resilient to chemotherapeutic treatments, is thought to be accountable for disease relapse, according to growing data. GCSC-like properties including drug resistance, self-renovation ability, and tumorigenicity were prevented in gastric cancer cell treatment with a lower dosage of genistein (15 M), which was linked to the extracellular signal-regulated kinase (ERK) 1/2 activity and inhibition of adenosine triphosphate binding cassette subfamily G member2 (ABCG-2) expression [79]. In GCSCs, genistein inhibits the Hedgehog signaling activator that is not only involved in oncogenesis but in cancer stemness, glioma-associated oncogene family zinc finger 1 (Gli1), and overexpression of CD44, a common GCSC surface marker too. According to CD44 expression, GCSCs sorted out from gastric cancer cell line of human, MKN45, were shown Gli1 and CD44 low expression on exposure to genistein. Furthermore, genistein inhibited CD44+ cells' strong cell migratory capacity, suggesting that it could be a useful drug for gastric cancer treatment by targeting cancer stem cell-like properties [80].

The article "Genistein: Therapeutic and Preventive Effects, Mechanisms, and Clinical Application in Digestive Tract Tumor" was published in 2022. Journal: Evid Based Complement Alternat Med.

In a concentration and time-dependent way, genistein dramatically reduced cell viability. On exposure of Gastric cancer cells to (0 M, 50 M, 70 M, and 90 M) Genistein had their p-38MAPK gene expression can lower up to 83%, 56%, and 57% respectively, and their cell proliferation decreased by percentage of 35, 52, and 67. Moreover, in treated cells, p-p38MAPK protein levels were much lower as compared to in untreated control cells. Genistein's varying dosages inhibited expression of the p38MAPK gene and growth of AGS stomach cancer cells as a promising option in therapeutic plant-derived drug of gastric cancer combination therapy [81]. Reference [82] found that genistein, a medication that inhibits KIF20A expression, has a stronger anticancer effect as compared to fluorouracil or cisplatin in gastric cancer, which could be useful in novel gastric cancer therapy development.

#### 2.6.3. *In Vivo* Studies

To improve the induction of stomach cancer, as an *In vivo* model, Wistar rats were injected with N-methyl-N′-nitro-N-nitroso guanidine and treated with NaCl [83]. They discovered that genistein's daily injections reduced vessel counts of the antral-mucosa, labeling index, and lowered the occurrence of stomach cancer after carcinogen treatment of 25 weeks, causing enhanced apoptosis and lowered angiogenesis of the stomach cancers.

From human gastric cancer cell line, MKN highly meta-static 85As2mLuc (2cachexia inducing sub-lines) and MKN45cl85 cell to examine the formation of malignant-progression of human stomach cancer and cancer cachexia. Cachexia is a common occurrence in mice when these two cell lines are used. In rats, long-term therapy with isoflavones resulted in tumor cytostasis, reduced cachexia, and longer survival (the anticancer impact was graded AglyMax > daidzein > genistein) [84]. Infection with *H. pylori* is linked to higher degrees of pro-inflammatory mediators (CINC-1 and TNF-), death of the gastric epithelial cell, and increased neutrophil permeation in the gastric mucosa. In rats with *H. pylori*-induced gastropathy, genistein reduced production of the pro-inflammatory cytokine, NF-kB initiation, and stomach apoptotic cell death, resulting in gastroprotection [85]. According to a study, in the indomethacin-treated rat, average serum TNF-alpha values were significantly higher as compared to the control group (210.28 0.98 vs. 126.4 0.13 pg/mL, *P*=0.001). In comparison to the indomethacin group, genistein caused a significant drop in stomach TNF-alpha levels (156.59 0.10 vs. 210.28 0.98 pg/mL, *P*=0.001) [86].

The article "Genistein: Therapeutic and Preventive Effects, Mechanisms, and Clinical Application in Digestive Tract Tumor" was published in 2022. Journal: Evid Based Complement Alternat Med.

To examine the genistein's protective effect, an experimental model of indomethacin-induced stomach damage was used. Before inducing stomach damage with indomethacin (50 mg/kg), genistein (10 mg/kg) was orally administrated for 7 days once daily. The stomach was taken out for biochemical and histological investigation. When compared to the indomethacin group, genistein dramatically reduced myeloperoxidase activity, malondialdehyde, tumor necrosis factor levels, and downregulating matrix metalloproteinase9 (MMP-9) gene expression [87].

### 2.7. Mechanisms and Clinical Application in Colorectal Cancer

#### 2.7.1. *In Vitro* Studies

In an advanced stage, colorectal cancer (CRC) is a fatal tumor that has a high degree of invasiveness and metastasis [88]. Numerous *in vitro* investigations have demonstrated that genistein has anti-cancer qualities against CRC and the methods by which it does so have been extensively studied. Genistein effectively by inhibiting the PI3K/Akt pathway inhibits colon cancer cell growth [89, 90], which plays a vital role in colon cancer progression regulation. ERs expression and tumor-suppressor genes in colon cancer cells are also impacted by genistein [91, 92]. It can suppress the Wingless and Integration-1 signaling pathways in the DLD-1 cell line, preventing uncontrolled cell proliferation [93]. In an SW480 human colon cancer cell line, genistein increased gene expression of Dickkopf-related protein 1 (DKK1), a Wnt signaling pathway antagonist, by inducing histone acetylation at the promoter region [94].

PEGylated silica hybrid nanomaterials of genistein cause the production of H_2_O_2_ and modulation of the antioxidant enzyme. The genistein nanomaterials start their antiproliferative and antioxidant activity on human colon cancer cell lines (HT29) and activate apoptosis and autophagy, unlike free genistein which only activates apoptosis in a low quantity [46]. In colon cancerous cells and tissues, CpG islands methylation in the promoter region decreased Wnt inhibitory factor 1 (WIF1) production. By demethylating WIF1, genistein restored WIF1 expression in the colon cancerous cells (HT29) and inhibited tumor cell migration and invasion. The foregoing findings could be linked to the control of migrating genes such as MMP2, MMP9, E-cadherin, TIMP1, -catenin, cyclin D1, c-Myc, and cell invasion [95]. It has been shown that genistein has antiproliferative properties that help to suppress CRC cells. These CRC cases had higher amounts of long noncoding RNA (lncRNA) TTTY18 expressions in a human study and transforming growth factor beta-1 (TGF-1), as well as upregulated serum and glucocorticoid regulated kinase-1 (SGK1), Ki-67, and Akt-Ser-473 expressions. Genistein-dosed CRC cells revealed lower cell viability, enhanced cell death, decreased Ki67 positive cells, decreased cell migration, and downregulated levels of SGK1, TTTY18, AktSer473, and p38 MAPKTyr323 *in vitro* [96]. The anticancer activities of chitosan encapsulated genistein were investigated. The CHI-En/Gen significantly slowed the growth and division of CRC cells in humans HT29. In HT-29 cells, caspase-3 gene expression analysis and flow cytometry demonstrated apoptotic cell death [97]. In CRC, genistein HCT-116 cells therapy resulted in induction of apoptosis and suppression of cell growth. Meanwhile, in HCT-116 cells, genistein reduced Akt, SGK1, and miR-95 mRNA levels and blocked Akt phosphorylation [98].

The article "Genistein: Therapeutic and Preventive Effects, Mechanisms, and Clinical Application in Digestive Tract Tumor" was published in 2022. Journal: Evid Based Complement Alternat Med.

Reference [99] evaluated the effect and mechanism of genistein on colon cancer cells' epithelial–mesenchymal transition (EMT) (HT-29 cells). Genistein impeded cell migration at 200 mol/L. Upregulation of E cadherin and downregulation of N cadherin, as well as repression of EMT-related makers, i.e., Snail2/slug, FOXC1, FOXC2, ZEB1, ZEB2, and TWIST1, reversed EMT in colon cancer cells. Furthermore, the expression of notch1, p-NFB, and NFB in HT29 cells is also inhibited by genistein, while Bax/Bcl2 and caspase3 expression is promoted. Pathways involving apoptosis and epithelial–mesenchymal transition (EMT) affected by genistein in HT29 cell lines are shown in Figure 2.

#### 2.7.2. *In Vivo* Studies

*In vivo* study revealed that using azoxymethane as a chemical inducer in case of colon cancer in male Sprague Dawley rats were treated with 140 mg genistein/kg body weight from gestation period to 13 weeks of age has shown a reduction in total aberrant crypts and a downregulation of Wingless and integration-1-catenin signaling, confirming this isoflavone preventing role [100]. In an *In vivo* investigation, genistein-dosed tumor-bearing nude mice had a decreased tumorous TGF-1 and TTTY18 concentration, as well as a lower body mass. Furthermore, the number of SGK1-, AktSer473-, and p38 MAPKTyr323-positive cells within the cell was reduced dose dependently. Overall, our human and experimental studies suggest that pharmacologically genistein exerts potential antimetastatic CRC benefits, presumably by blocking the TTTY18/Akt pathway in CRC cells through a molecular mechanism [96]. Genistein dramatically slowed the growth of a mouse xenograft tumor in CRC mice *in vivo* [98]. In high-fat mice, a genistein-rich diet was tested for its ability to prevent azoxymethane/dextran sulfate sodium (AOM/DSS)-induced colon cancer. In comparison to the control group, genistein supplementation can help prevent colon cancer. In the genistein-treated group, the expression of COX2, TNF, and FRAT-1 mRNA was reduced. In addition, a genistein-rich diet has been shown to reduce colon cancer viability through modulating the expression of PI3K, AKT, and FOXO3. Genistein has been demonstrated to inhibit the formation of colonic neoplasms via regulating the PI3K/FOXO3/AKT signaling mechanism, in mice fed with a high-fat diet [101].  Figure 3 highlights the apoptotic role of genistein in colorectal cancer by inhibiting different pathways.

The article "Genistein: Therapeutic and Preventive Effects, Mechanisms, and Clinical Application in Digestive Tract Tumor" was published in 2022. Journal: Evid Based Complement Alternat Med.

*Fructus sophorae* genistein (FSGen) has been demonstrated to have bioactivity in the treatment of radiation-induced intestinal damage. In a study, C57/BL mice were given 7.5 Gy whole-body irradiation with FSGen therapies. After irradiation, tissue investigation revealed considerable structural and functional recovery of the gut in FSGen-pretreated cohorts. A study showed that IEC6 cells are protected by FSGen from radiation injury by upregulating the Rassf1a and Ercc-1 genes to successfully weaken DNA irradiation injury using protein expression, mRNA expression, and small interfering RNA analysis [102]. In genistein-treated tumor transplanted nude mice, tumor development was reduced, which was followed by dose-dependent downregulations of KDR proteins, MCL1, APP, and mRNAs [103].

## 3. Conclusion and Future Perspective

This study paper conducted an in-depth assessment of the scientific literature on the possible function of genistein as an antigastrointestinal cancer agent before publishing it. Using genistein therapy for cancer treatment in underdeveloped nations, where currently available cancer treatments are prohibitively expensive, has the potential to be highly effective. The use of natural ingredients for cancer therapy appears to have promise in terms of cost-effectiveness. Genistein (an isoflavone) is a natural chemical that has bioactive properties. The clinical and experimental data obtained in this paper demonstrate that genistein is involved in a wide variety of carcinogenic molecular pathways, indicating that it has great therapeutic potential in the treatment of cancer. As a result, synergistic methods based on genistein may be beneficial soon for cancer therapy.

The article "Genistein: Therapeutic and Preventive Effects, Mechanisms, and Clinical Application in Digestive Tract Tumor" was published in 2022. Journal: Evid Based Complement Alternat Med.

To fully understand the chemo-preventive and therapeutic potential of genistein, large patient cohorts will be necessary to conduct clinical research. The drug–drug interactions of genistein with other chemotherapeutic drugs require more investigation. Genistein's accessibility and bioavailability must be increased, and it is necessary to investigate the mechanisms and techniques that may be used to do this. It is necessary to standardize the precise therapeutic dose of genistein (as well as the length and timing of genistein dose administration) for the treatment of various GI cancers. Additionally, the function of nanotechnology should be investigated to minimize the number of doses necessary and to more specifically target tumor tissues using new drug delivery methods.

## Figures and Tables

**Scheme 1:** Deoxybenzoin route of genistein synthesis using DMF/PCl_5_ as a source of (Me_2_N = CHCl)C_l0_ [26].

**Scheme 2:** The chalcone method of genistein synthesis [26].

**Figure 1:** The anti-cancer effect of genistein: downregulating/suppressing, inhibiting, and enhancing different pathways. AP-1; Bax; Bcl-2; EGFR; I*κ*B; KIF20A; PI3K/Akt; TRAIL; TRAIL R; Wnt1/*β*-catenin modified from [21].

**Figure 2:** Pathways involving, apoptosis and epithelial–mesenchymal transition (EMT) effect by genistein in HT29 cell lines. EMT reverses genistein by enhancing the expression of E-cadherin and inhibition of N-cadherin; along with the control of ZEB1, EMT makers, TWIST1, and Snail2/slug. Genistein enhances the function of Bax/Bcl-2 and caspase-8 by impeding notch-1. A decrease in the notch-1 leads to the prevention of both NF-*κ*B and p-NF-*κ*B expression, resulting in EMT reduction. Adapted and modified from [99].

**Figure 3:** The pathways involved in colon cancer inhibited by genistein. Adapted and modified from [101].

**Table 1:** Summary of genistein's usage against cell lines of cancer other than gastrointestinal cancer.

Cancer type	Cell line used	References
Thyroid carcinoma	CAL-62, ACC 448	Ozturk et al. [53]
Pancreatic carcinoma	Mia-PaCa2 and PANC-1	Bi et al. [54]
Breast cancer	MCF-7, SK-BR-3, MDA-MB-231 and ZR-75-1	Chen et al. [55, 56]
Esophageal carcinoma	Eca-109, EC9706 and CaES-17	Gao et al. [57]
Liver cancer	Hep-G2, SMMC7721, and Bel7402, Hep-3B, HuH7	Chodon et al. [58–62]
Prostate cancer	LNCaP, DU-145 and PC3	Li et al. [63–67]
Lung cancer	A-549, Calu-1, H-1975, and NCL-H460	Zhang et al. [68]
Cervical cancer	HeLa and CaSki cells	Liu et al. [69]
Ovarian carcinoma	SKOV3, OVCAR-5	Huang et al. [70, 71]

The article "Genistein: Therapeutic and Preventive Effects, Mechanisms, and Clinical Application in Digestive Tract Tumor" was published in 2022. Journal: Evid Based Complement Alternat Med.

## Data Availability

This article does not contain any additional data.
